RETRACTED

# Perceived Security Risk Based on Moderating Factors for Blockchain Technology Applications in Cloud Storage to Achieve Secure Healthcare Systems

**DOI:** 10.1155/2022/6112815

**Published:** 2022-01-19

**Authors:** Malik Mustafa, Marwan Alshare, Deepshikha Bhargava, Rahul Neware, Balbir Singh, Peter Ngulube

**Affiliations:** ^1^Faculty of Computing Sciences, Gulf College, Muscat, Oman; ^2^DIT University, Dehradun, India; ^3^Department of Computing, Mathematics and Physics, Høgskulen på Vestlandet, Bergen, Norway; ^4^Administrative Staff College of India, Hyderabad, India; ^5^Malawi University of Science and Technology, Malawi

## Abstract

Due to the high amount of electronic health records, hospitals have prioritized data protection. Because it uses parallel computing and is distributed, the security of the cloud cannot be guaranteed. Because of the large number of e-health records, hospitals have made data security a major concern. The cloud's security cannot be guaranteed because it uses parallel processing and is distributed. The blockchain (BC) has been deployed in the cloud to preserve and secure medical data because it is particularly prone to security breaches and attacks such as forgery, manipulation, and privacy leaks. An overview of blockchain (BC) technology in cloud storage to improve healthcare system security can be obtained by reading this paper. First, we will look at the benefits and drawbacks of using a basic cloud storage system. After that, a brief overview of blockchain cloud storage technology will be offered. Many researches have focused on using blockchain technology in healthcare systems as a possible solution to the security concerns in healthcare, resulting in tighter and more advanced security requirements being provided. This survey could lead to a blockchain-based solution for the protection of cloud-outsourced healthcare data. Evaluation and comparison of the simulation tests of the offered blockchain technology-focused studies can demonstrate integrity verification with cloud storage and medical data, data interchange with reduced computational complexity, security, and privacy protection. Because of blockchain and IT, business warfare has emerged, and governments in the Middle East have embraced it. Thus, this research focused on the qualities that influence customers' interest in and approval of blockchain technology in cloud storage for healthcare system security and the aspects that increase people's knowledge of blockchain. One way to better understand how people feel about learning how to use blockchain technology in healthcare is through the United Theory of Acceptance and Use of Technology (UTAUT). A snowball sampling method was used to select respondents in an online poll to gather data about blockchain technology in Middle Eastern poor countries. A total of 443 randomly selected responses were tested using SPSS. Blockchain adoption has been shown to be influenced by anticipation, effort expectancy, social influence (SI), facilitation factors, personal innovativeness (PInn), and a perception of security risk (PSR). Blockchain adoption and acceptance were found to be influenced by anticipation, effort expectancy, social influence (SI), facilitating conditions, personal innovativeness (PInn), and perceived security risk (PSR) during the COVID-19 pandemic, as well as providing an overview of current trends in the field and issues pertaining to significance and compatibility.

RETRACTED

## 1. Introduction

Because healthcare is such a vital part of everyone's life, it has become critical to diagnose patients and store them for future reference to secure healthcare data such as drugs and past health records. Initially, this medical data was meticulously transcribed into electronic form from paper records. There were numerous opportunities to alter and corrupt the data when using this method. As a result, electronic storage of healthcare data is crucial. Healthcare databases, on the other hand, run the possibility of being irreversibly altered or deleted, and data blocking is also a concern. Whenever medical data that should not be available to anybody other than patients or hospitals is obtained by an unintended entity like a person, a data blockage occurs. It is possible for technology to improve people's quality of life by addressing resource allocation and information blockade issues. For cloud-based healthcare data sharing, it is all about timing. References [1–3] are possible answers. There are several privacy and security concerns when it comes to cloud computing despite its popularity and numerous offerings [2–6]. Global organizations have focused on developing security rules and processes for the cloud environment before using it for their business solutions as a result of this [7–11]. As a result, cloud service providers can no longer afford to lose their clients' confidence in the security and privacy of their outsourced data. Its limits make distributed and decentralized security measures more important in a cloud context.

It is widely believed that blockchain (BC) technology is the best way to provide security to cloud infrastructure [12–16] because of the distributed network's interconnectedness and the cloud's importance. Blockchain technology may be the best secure solution for a cloud environment because of its ability to communicate quickly and demand substantially fewer processing resources. In other words [10], by utilizing blockchain technology's inherent security, once transaction information has been recorded and updated, they can no longer be changed or deleted. The distributed data ledger can support exceptional immutability and data security even though it is shared across all nodes in the cloud [17–19]. Because of the employment of cryptographic algorithms in the blockchain blocks, the privacy of the data is more likely to be protected. Because of these features, the blockchain is the most likely candidate to deliver cloud data security. According to the findings of this study, blockchain technology can be used in the cloud for secure transmission of healthcare data [20–23]. The health sector is a major concern for both developing and developed countries, as this sector is directly related to people's social well-being and life. The security of such crucial data is important to avoid the privacy leaks. It will thus improve the healthcare system, and e-health records will be a huge aid in taking care of patients. Research and development in the health sector should be an ongoing process as it will help improve the quality of life by combating various health problems and diseases.

RETRACTED

## 2. Cloud Security Systems

Medical data concerning patients' ailments or past medical records must be precisely captured and stored and shared securely in order to maintain the privacy of patients' private information in the creation of smart hospitals. A totally trustworthy server is required in the old method of controlling data access, which makes it difficult to adapt to today's scattered network environment. A new viewpoint on end-to-end communication, encryption methods, consensus mechanisms, and distributed data storage has been provided by blockchain because of its decentralization and security. Since then, ABE (attribute-based encryption) has become a crucial solution for satisfying cloud security needs. In addition, the ABE cloud access control mechanism has been thoroughly examined [24–27], respectively. It is important to have some way of connecting users to the encrypted data because an attribute-based encryption system uses public keys as attributes. Cloud data storage security is greatly enhanced by its configurable encryption and access control features. In the meantime, it has evolved into a critical method for securing cloud data storage. It also enables more granular control over access. However, the classic ABE does not fully ensure data privacy, effective collision prevention, or assurance of attribute revocation-based forward and backward security. Revocation has also resulted in significant computing costs [18, 28, 29], respectively. In order to increase data storage security and cloud computing performance, implementing blockchain technology and its security measures will become a critical study area. The mismatch between data privacy and data sharing can be remedied by combining blockchain and cloud computing, as well as a strong security methodology [30–33].

RETRACTED

### 2.1. Existing Cloud Security System Limitations

As stated in the preceding section, the majority of security solutions deployed in the cloud do not have a distributed character. Cloud computing, on the other hand, is a distributed system; therefore data is dispersed over the cloud as well. As a result, it is critical to use contemporary cloud computing security methods. In addition, not all security systems are as open and accessible as others. Due to current security methods, data is very changeable, suggesting that each node can easily alter it. There are now resource-intensive and expensive security solutions in place [34].

### 2.2. Research Problem of Blockchain

Recent years have seen a lot of work done on blockchain technology. As a backend for the digital currency Bitcoin, blockchain technology was initially created [35]. In the same way that contemporary cloud computing provides a framework for collaboration among strange and unreliable entities, the blockchain technology's core model is akin to that. Mobile or intelligent health device features can be provided without a central authority for security and authentication. A “public-ledger” data record serves as the foundation for this system, which is accessible to all participants. A block of data linked to the use of a cryptographic hash key can be found in this public-ledger record. This method of reaching agreement or connection is known as proof of work (PoW). Data manipulation has no effect on agreement or ledger because they are naturally independent. By canceling prior Blockchain block hashes, the block data breaches the consensus among nodes and must be removed. After the fact, it cannot be changed. Anticipation, effort expectations, social influence (SI), facilitation factors, personal innovativeness (PInn), and a perception of security risk have all been proven to influence blockchain adoption (PSR). During the COVID-19 pandemic, anticipation, effort expectancy, social influence (SI), facilitating conditions, personal innovativeness (PInn), and perceived security risk (PSR) were found to influence blockchain adoption and acceptance, in addition to providing an overview of current trends in the field and issues pertaining to significance and compatibility.

### 2.3. Background Research on the Blockchain

Previously, the blockchain was restricted to the financial industry, but it now includes a wide range of other applications, including public healthcare. One of the most promising areas of recent research has been blockchain-based medical solutions. There should be no tampering with the medical data that is collected. Anyone who wants the data should be obliged to confirm its accuracy, be it the researcher, the patient, the patient's family, or anyone else. In order to communicate data securely, academics have attempted to combine blockchain technology with other technologies. Multiple researchers utilized the blockchain to merge various technologies. In the agro-food supply chain monitoring sector, one of these regularly utilized technology applications is RF identification with blockchain [36]. Other uses for blockchain include IoT, the automotive industry, and smart contracts. Blockchain technology has a wide range of potential applications.  Figure 1 shows an example of a typical blockchain diagram.

RETRACTED

## 3. Blockchain Security in Healthcare System Survey

### 3.1. Smart Healthcare and Blockchain

It was determined that blockchain technology might be used in smart healthcare systems as part of this study. Throughout the last few decades, healthcare systems have been increasingly concerned about cyber dangers. Patients' privacy and security are jeopardized because of the lack of adequate infrastructure for protecting medical data from data breaches of this nature. Health organizations now have control over patient data, putting the privacy of that data at risk and making it difficult to exchange information about a patient's treatment. Because of the potential for treatment delays, transferring patient health information from one service provider to another requires more time. Blockchain technology has the potential to assist EHR in overcoming these real-world obstacles. Several businesses, governments, and public-private partnerships have recently turned to blockchain technology. A focus by the FDA and IBM Watson Health to preserve oncology-related data made the benefits of blockchain technology in the healthcare sector evident [37].

This blockchain's transaction audit log can store data gathered from a variety of sources. As time goes on, this transaction audit record will be useful for tracing the ownership and transparency of data as it is exchanged. The FDA and IBM claim that the blockchain can aid in data interchange by assessing multiple data gathering sources with patient consent and terms that are mutually agreed upon. There is a current model based on secret data being transported and stored on the cloud, which is not secure or dependable at this time. Access to healthcare data must also be handled with care. Maintaining data integrity has mandated standard auditing in the same way. Data integrity, anonymity, secure storage, and less likelihood of data infringement are all provided by the blockchain. Additionally, because of the distributed nature of blockchain technology, the risk of a single point of failure is decreased [38].

RETRACTED

### 3.2. In Healthcare, Blockchain Is Used with Cloud Computing

There are numerous issues raised by smart hospitals regarding secure health data sharing and patient privacy protection, so this study focuses on a blockchain-based distributed healthcare data privacy protection strategy combined with a cloud computing-based distributed healthcare data privacy protection strategy Or to put it another way, a distributed blockchain-based data management architecture for smart hospitals is being developed, with a cloud computing paradigm and a distributed blockchain-based data management architecture designed exclusively for them. Consumers can get specific access control systems by using encryption and proxy reencryption and ABE technologies to deal with the high computational costs. Patients' healthcare information can be sent securely between doctors using status and attribute-based user access. This response's entire healthcare data is encrypted at the bottom. Cloud nodes process the transferred healthcare data and return the final ciphertext on the request side after it has been received and processed by the nodes. Instead, proxy reencryption and data sharing with privacy limits enforced by the cloud environment's service side are meant to deal with issues of safe data storage and exchange primarily among smart hospitals [17, 39, 40].

### 3.3. EMR, EHR, or PHR Ecosystem Based on Blockchain

For the purpose of this essay, the inner workings of a blockchain-based electronic medical records, electronic healthcare records, or personal health record ecosystem were examined. Using blockchain technology, which is well-known for its successful application in Bitcoin, to secure healthcare data management, has recently piqued public interest. An open-ended and distributed online database can be created using blockchain technology, which uses data blocks, such as lists of data structures that are linked to one another so that each block refers to the one before it. Infrastructure nodes spread such collaborations rather than keeping them in a centralized storage facility. Patients' healthcare data and healthcare provider details from our perspective are included in every block, as well as the timestamp of block generation and the hash of the previous block.  Figure 2 shows a hypothetical blockchain-based EMR, EHR, or PHR system (2). Once a new piece of healthcare data on an individual patient is created, a new block is generated and broadcast to all end nodes in the patient network. By adding a new block once it has been approved by most of the chain's end nodes, it will be possible to get an accurate, reliable, and efficient picture of a patient's medical history. A fork happens when the chain cannot agree, and the block is left as an orphan on the main chain. A new block cannot be added to the chain without also modifying the data in all previous blocks. There is no way to avoid this.

RETRACTED

On the other hand, change is easy to spot. Data on healthcare must be protected before it is presented in the block because it is publicly available. Because of its decentralized consensus and consistency, blockchain is theoretically impervious to deliberate and/or unintended attacks [41–44].

When a deal is reached without involving a trusted mediator, there will be no blockage or single point of failure. Patients will have control over their data, and healthcare information will be distributed as blockchain data in a consistent and complete manner. Changes in blockchain will be visible to all patients in the network, and all data insertions will be immutable.

## 4. Research Findings and Discussion

This part covers the following topics: respondent profile, exploratory factor analysis test (EFA), goodness, and construct validity fitness.

### 4.1. Profile of the Respondents

This study involved 443 research participants selected from Middle East countries, and these participants completed the online questionnaire.  Table 1 accordingly displays the participants' personal information.

It can be observed in Table 1 that more than half (55.1%) of the respondents involved in virtual reality training were male, and the majority of respondents, or 38.0%, were between the age of 20 and 30. About one-fourth of the respondents were between the age of 31 and 41, while 22.2% were between 42 and 52, whereas the remaining 14.8% were above 53 years of age. The following are the students' virtual reality learning results. A whopping 12.0% of respondents said they had “no prior experience.” A total of 19.3 percent of respondents said they had 1 to 2 years of experience, 19.0 percent said they had 3 to 4 years of experience, 17.5 percent said they had 5 to 6 years of experience, 14.8 percent said they had 6 to 7 years of experience, and 17.4 percent said they had more than 8 years of experience. The results in the table show the following information about respondents' educational backgrounds: 14.3 percent stated they had just completed elementary school, 19.4 percent said they had completed high school, 31.7 percent said they had completed college, and 35.3 percent said they had completed a university education.

RETRACTED

The construct validity of all variables was assessed using factor analysis, and the sample size score was used to gauge the study's trustworthiness. The sample was analyzed and reevaluated using a dependability test. Cronbach's alpha was used to assess the major variables' internal consistency. The scale's dependability was evaluated through an iterative process as well. If removing an item off the scale makes it more reliable, that will be investigated. Objects that fail this test are discarded and the test is redone. Since the sample size was very big, we used quantitative analysis tools and different tests in order to obtain accurate data and results. The data was collected of both the genders of varying age group from different sectors.

### 4.2. Analyze the Data

SPSS (Statistical Package for the Social Sciences) v13 was used to execute the analysis. The respondents' profiles were investigated using descriptive analysis, which included percentage and frequency tests. Pearson correlation analysis, independent *T*-test sample, chi-square independence test, and multiple linear regressions were among the other tests utilized in this study. The applied significance level was 5%.

#### 4.2.1. Validity of the Measures

SPLS (Smart Partial Least Squares) and SPSS (Statistical Package for the Social Sciences) were applied in this study to verify the study dimensions and test the entire framework of the proposed model. The discriminant and convergent validity were ascertained through factor analysis, and the details are provided in Table 2; all concepts scored above 0.80 for Cronbach's alpha.  Table 3 shows the result of factor analysis. On the other hand, Table 4 shows that the average variance extracted (AVE) score for all images is more significant than 0.75 (Table 4 diagonal elements), providing assurance that the AVE of each construct is more powerful compared to the squared relations between constructs.

Table 2 displays the results of the descriptive test on the general situation of Middle Eastern universities in terms of standard deviation, mean, minimum, and maximum values. Furthermore, to make the 5-point Likert scale easier to comprehend, scores greater than 3.67 (highest value (5)-4/3) were considered high, scores less than 2.33 (4/3 + lowest rate (1)) were labeled soft, and moderate.

The modest rise in results was not eliminated, as suggested by [10], because it was unnecessary, given that, as shown in Table 2, the alpha values for all variables in this sample are more significant than 0.7. Table 2 shows the 29 items used in this study, as well as the results of many regular reliability checks. As a result, the most tiny Cronbach's alpha score for dependability is 0.726, according to the item statistics. To put it another way, the constructs are generally reliable.

RETRACTED

#### 4.2.2. The Partial Least Squares Method Is Used to Solve Problems

The partial least squares (PLS) method is a two-step method that produces a smaller collection of different components from a large number of predictors. The use of the PLS technique is appropriate for a small sample [36]. If there are formative constructs, each question must have 10 responses for the sample size for PLS, as stated by [37]. Additionally, evaluating model measurement's acceptability [37] requires evaluating item reliability, internal consistency, and discriminant validity. This study employed 40 items representing five dimensions, and Smart PLS software was used to test these items.  Table 1 presents the details.

Furthermore, the item loadings were chosen to determine the individual things' dependability, and it is critical that the item loadings carry good value or they will be withdrawn from their respective constructs. Ref. [38] advised that the items have a minimum loading value of 0.3 to be considered relevant.

Given that items with a loading value of 0.4 were considered significant, complete items with loading values greater than 0.5 were deemed very significant. As a result, a threshold value of 0.4 was used as a criterion for item acceptability for the specified dimensions in this investigation. The model obtained loading values above 0.4 for all items of all sizes in this sample. Each item's *t* value was larger than 2.58; hence, they were all regarded significant in terms of their constructions.

Additionally, the minimum consistency score is 0.7, and the internal consistency of the latent variables was tested following [17]. Furthermore, the composite reliability (CR) and Cronbach's alpha results surpassed the thresholds. Lastly, all latent variables scored AVE greater than 0.

This study examined the discriminant validity of the latent variables, as suggested by [17]. The correlations between the other variables must be less than the square roots of AVE in this case. The integers in the off-diagonal of the matrix represent the correlations. The square root of AVE is used to represent the diagonal values in Table 4. In this case, AVE's square roots must be bigger than the correlations' values [37]. The results support the validity and discreteness of each latent variable as a construct.

Table 4 shows the general state of educational institutions in Middle Eastern countries as a result of descriptive study. The table shows the mean, lowest, and maximum values, as well as the standard deviation (S.td) of the variables, and the 5-point Likert scale is divided into three categories: scores of 2.33 and below (lowest rate 1) are considered weak, 3.67 and above (higher rate 5) are considered crucial, and scores in the middle are considered intermediate.

RETRACTED

The indirect and direct impacts of the discrete independent variable on behavioral intention are displayed in Tables 3 and 4. As shown, all hypotheses were supported, with the exclusion of hypotheses H4 and H5—Table 3 can be referred to. Notably, as can be viewed in Table 5, the model proposed in this study explained 73% of the variance in personal innovativeness, 62% of the variance in perceived security risk, and 70% of the variance in behavioral intention.

Concerning the analysis, it can be construed for H1 that perceived security risk (PSR) directly affected behavioral intention (BI), while for H2 the result shows that personal innovativeness (PInn) affected behavioral intention (BI) over gender. The result for H3 shows that effort expectancy directly affected behavioral intention (BI). In contrast, for H4, the result shows that social influence directly did not affect behavioral intention (BI). For H5, the result shows that performance expectancy directly did not affect behavioral intention (BI) over gender. As for H6, the result proves that facilitating conditions directly affected use behavioral (UB) over gender.

Further, the results show support to hypotheses H7, H9 to H17, and H18. On the other hand, hypothesis H8 was not supported. The obtained results denote either indirect or direct impact of all model variables on behavioral intention. As shown in Table 6, the results led to the conclusion of a significant relation between behavioral intention and perceived study risk.

Based on the data, it can be concluded that the availability of infrastructure and the security of healthcare systems in Middle Eastern nations have hampered the spread of blockchain technology. Meanwhile, the current students' basic understanding of blockchain technology is investigated in this study, and the findings show that students are reasonably aware of the limitations of blockchain technology.

When studying user behavior, it is critical to know what students think about blockchain technology and how it relates to healthcare security. Students' intents to use blockchain technology had a positive impact on user behavior, even though the *R*^2^ score was minimal.

### 4.3. Result Summary

A set of data gathering is used to assess the performance of the blockchain approach. Each work uses a similar dataset to obtain reliable and consistent results by checking the time spent accessing the EHR and the processing time complexity. Electronic health records (EHRs) from individual patients are included in the experiment's dataset; however, this information should not be disseminated. Healthcare providers, insurers, and competitors may profit from exploitation of patient personal information, such as medical, treatment, and financial data. With this dataset, researchers can analyze and validate the processing time and temporal complexity of various cloud technologies, including those that use authentication mechanisms such as blockchain and/or the distributed ledger technology (DLT).

RETRACTED

Figure 3 compares the amount of time required to use the various technologies examined throughout this study. It is inevitable from the graph of Figure 3 that for a particular size, the time taken by block and cloud computing is less compared to that by the other intelligence platforms. Thus, it is clear that blockchain technology deployed with cloud storage helps to improve healthcare system security. For example, blockchain and the cloud integrated with blockchain technology have a lower time consumption with increasing file size when processing EHR data than traditional cloud computing and the cloud combined with authentication technologies. As a result, blockchain technology is superior to the rest.

Meanwhile, Figure 4 depicts the temporal complexity achieved by different strategies in terms of processing time. The temporal complexity of blockchain technology and blockchain technology integrated cloud is lower than the other two standard cloud-based technologies. So, it is clear from Figure 4 that blockchain could reinvent the way in which patient electronic health records are shared and stored, by providing more secure healthcare information exchange mechanisms in the healthcare sector and securing them over a decentralized peer-to-peer network.

In addition, as shown in Table 7, the overall performance of these four technologies is reviewed and compared in terms of data accessibility and security characteristics.

## 5. Conclusion

Security and privacy issues are now a major concern for intelligent healthcare systems. To avoid such problems, it is vital to comprehend the security requirements of those systems. Intelligent healthcare systems now face a plethora of security and privacy concerns. It is critical to understand the security requirements of those systems in order to avoid such issues. There was also some fear of data suffocation. Some efforts concentrating on healthcare data security using blockchain technology, as well as relevant research, are examined in this paper. This research also looks at the privacy and storage security issues that exist in the cloud. Then, it was discovered that blockchain technology exceeds conventional technologies in terms of security efficiency and efficacy. This study looked into a variety of elements that influence the adoption of blockchain technology in Middle Eastern countries' innovative healthcare systems.

RETRACTED

The impact of personal creativity and its relationship to behavioral intent were also explored. The impact of individual innovation considerations on the adoption of blockchain technology for innovative healthcare systems in Middle Eastern countries was also investigated. This has a direct bearing on the deployment of blockchain technology in the outstanding healthcare systems of these countries. Given the aforementioned, the study looked into the power of demographic characteristics as moderators. As a result, future research might consider gender, age, and knowledge with blockchain technology, as well as their impact on blockchain adoption for smart healthcare systems. Another research topic for the future is to investigate all of the elements that influence blockchain technology acceptance. The findings of this study revealed a lack of understanding of the primary influencing factors when it comes to implementing blockchain technology in these countries' healthcare services and technology. When studying user behavior, it is critical to know what students think about blockchain technology and how it relates to healthcare security. Students' intents to use blockchain technology had a positive impact on user behavior, even though the *R*^2^ score was minimal. Future research might consider gender, age, and knowledge with blockchain technology, as well as their impact on blockchain adoption for smart healthcare systems. Another research topic for the future is to investigate all of the elements that influence blockchain technology acceptance.

## Figures and Tables

**Figure 1:** Typical blockchain diagram.

**Figure 2:** Blockchain-based EMR, EHR, or PHR conceptual ecosystem.

**Figure 3:** Time consumption for electronic health record access.

**Figure 4:** Time complexity comparison graphs with respect to processing time.

**Table 1:** Profile of respondents (*N* = 443).

Measure	Item	Frequency	Percentage (%)	Cumulative %
Gender	Male	244	55.1	55.1
	Female	199	44.9	100
Age	20-30	167	37.7	37.3
	31-41	111	25.1	62.4
	42-52	99	22.2	84.6
	53 and above	67	15.0	100
Experience	No experience	60	13.5	13.5
	1–2 years	79	17.8	31.3
	3–4 years	86	19.4	50.7
	5–6 years	81	18.3	69.0
	6–7 years	65	14.7	83.7
	8–above	70	16.3	100
Educational background	Elementary school	75	16.9	16.9
	High school	88	18.9	35.8
	College degree	129	30.1	65.9
	Graduate degree	151	34.1	100
Total		443	100%	

RETRACTED

**Table 2:** Cronbach's alpha test results of the framework study.

Constructs	No. of item	AVE	Alpha
Perceived security risk (PSR)	5	0.94	0.731
Performance expectancy (PF)	4	0.92	0.771
Effort expectancy (EE)	3	0.86	0.775
Social influence (SI)	4	0.87	0.771
Facilitating conditions (FC)	4	0.86	0.726
Personal innovativeness (PInn)	3	0.84	0.762
Behavioral intention (BI)	3	0.85	0.751
Use behavior (UB)	3	0.91	0.771

**Table 3:** The result of factor analysis.

Variables	Dimensions	Factor loading (FL)	Mean ± SD	Composite reliability (CR)	Cronbach's alpha	Average variance extracted (AVE)
Perceived security risk (PSR)	PSR1	0.758	3.755 ± 0.936	0.874	0.717	0.632
	PSR2	0.738	3.776 ± 0.834			
	PSR3	0.878	3.753 ± 0.723			
	PSR4	0.796	3.741 ± 1.083			
	PSR5	0.856	3.753 ± 0.723			
Performance expectancy (PF)	PF 1	0.738	3.767 ± 1.071	0.865	0.858	0.653
	PF 2	0.753	3.763 ± 1.041			
	PF 3	0.738	3.767 ± 1.029			
	PF 4	0.726	3.853 ± 0.775			
Effort expectancy (EE)	EE1	0.753	3.797 ± 1.021	0.768	0766	0.672
	EE2	0.796	3.752 ± 1.081			
	EE3	0.874	3.734 ± 1.031			
Social influence (SI)	SI1	0.833	3.875 ± 0.981	0.727	0.958	0.841
	SI2	0.742	3.744 ± 0.764			
	SI3	0.776	3.872 ± 0.854			
	SI4	0.857	3.738 ± 1.026			
Facilitating conditions (FC)	FC1	0.768	3.854 ± 1.062	0.876	0.853	0.785
	FC2	0.761	3.834 ± 0.731			
	FC3	0.857	3.825 ± 0.889			
	FC4	0.816	3.734 ± 0.865			
Personal innovativeness (PInn)	PInn1	0.718	3.821 ± 0.873	0.877	0.862	0.734
	PInn2	0.715	3.835 ± 0.853			
	PInn3	0.829	3.657 ± 1.835			
Behavioral intention (BI)	BI1	0.738	3.739 ± 0.764	0.872	0.846	0.645
	BI2	0.866	3.724 ± 0.774			
	BI3	0.754	3.872 ± 0.854			
Use behavior (UB)	UB1	0.821	3.754 ± 0.754	0.862	0.858	0.766
	UB2	0.853	3.872 ± 0.874			
	UB3	0.723	3.738 ± 1.026			

**Table 4:** Descriptive statistics analysis, reliability factors (*α*), and correlations (*N* = 432).

Constructs	*M*	SD	1	2	3	4	5	6	7	*α*
PSR	3.786	3.532	0.77	0.56^∗∗^	0.65^∗∗^	0.56^∗∗^	0.35^∗∗^	0.72^∗∗^	0.35^∗∗^	0.74
PE	3.782	3.542		0.57^∗∗^	0.45^∗∗^	0.55^∗∗^	0.34^∗∗^	0.75^∗∗^	0.34^∗∗^	0.75
EE	3.765	3.785			0.32^∗∗^	0.54^∗∗^	0.39^∗∗^	0.66^∗∗^	0.39^∗∗^	0.81
SI	3.787	3.734				0.62^∗∗^	0.58^∗∗^	0.56^∗∗^	0.35^∗∗^	0.72
FC	3.765	3.834					0.62^∗∗^	0.69^∗∗^	0.72^∗∗^	0.75
PI	3.789	3.734						0.52^∗∗^	0.46^∗∗^	0.76
BI	3.712	3.657							0.56^∗∗^	0.91
UB	3.783	3.821								0.73

**Table 5:** Results of the hypotheses' tests (direct effects on behavioral intention).

Hypothesis	Relationship	Path coefficient	Standard error	*t* value	Supported	
H1	Perceived security risk➔behavioral intention	1.368	0.121	2.971	∗∗∗	Yes
H2	Personal innovativeness ➔ behavioral intention	0.312	0.094	0.154	∗∗	Yes
H3	Effort expectancy ➔behavioral intention	0.595	0.052	1.702	∗	Yes
H4	Social influence➔ behavioral intention	-0.396	0.043	10.334	n.s	No
H5	Performance expectancy ➔behavioral intention	-1.021	0.148	7.011	n.s	No
H6	Facilitating conditions ➔use behavior	0.668	0.115	1.583	∗∗∗	Yes

RETRACTED

**Table 6:** Hypotheses' results (indirect effects on behavioral intention (BI)).

Independent	Mediator	Dependent	Hypothesis	*T*	Sig. (*p*)
PSR	Gender	BI	H7	1.574	Yes^∗∗^
PE	Gender	BI	H8	-2.210	No
EE	Gender	BI	H9	1.325	Yes^∗∗^
SI	Gender	BI	H10	0.873	Yes^∗^
PInn	Gender	BI	H11	1.514	Yes^∗^
FC	Gender	UB	H12	0.368	Yes^∗^
PSR	Experience	BI	H13	1.324	Yes
PE	Experience	BI	H14	-1.162	Yes^∗^
EE	Experience	BI	H15	0.992	Yes^∗∗^
SI	Experience	BI	H16	0.472	Yes^∗^
PInn	Experience	BI	H17	-1.142	Yes
FC	Experience	UB	H18	0.865	Yes

**Table 7:** Comparison of performance analysis.

Properties	Cloud	Cloud with authentication	Blockchain	Cloud+blockchain
Flexibility	No	Low	High	Very high
Decentralized access	No	No	Yes	Yes
Integrity	Yes	Yes	Yes	Yes
Data privacy	Less	Medium	High	Very high

## Data Availability

The data used to support the findings of this study are available from the corresponding author upon request.
